The article "Spiral Computed Tomography in the Quantitative Measurement of the Adjacent Structure of the Left Atrial Appendage in Patients with Atrial Fibrillation" was retracted in 2023. Reasons: signs of a paper mill; suspected computer-generated content; unreliable results or conclusions; lack of ethics approval or compliance.

# Spiral Computed Tomography in the Quantitative Measurement of the Adjacent Structure of the Left Atrial Appendage in Patients with Atrial Fibrillation

**DOI:** 10.1155/2021/9893358

**Published:** 2021-11-30

**Authors:** Zhen Zhang, Wei Yan

**Affiliations:** Department of Cardiovascular Medicine, Affiliated Hospital of Youjiang Medical College for Nationalities, Guangxi Baise 533000, China

## Abstract

Cardiac arrhythmias are common clinical cardiovascular diseases. Arrhythmias are abnormalities in the frequency, rhythm, site of origin, conduction velocity, or sequence of excitation of the cardiac impulses. Arrhythmia mechanisms include foldback, altered autonomic rhythm, and triggering mechanisms. It can cause palpitations, dizziness, black dawn, syncope, and angina pectoris and can worsen a preexisting cardiac disease, reduce the quality of life, and increase mortality. Also, by making it one of the constant challenges for the clinical cardiovascular physician, we can get more information. The study included 94 patients with atrial fibers, including 56 men and 38 women aged 57, 46, 11, and 68 years. There are 80 patients with nonatrial fibers, including 44 men and 36 women aged 56, 10, and 83 years. Those who can perform a normal coronary angiography and exclude congenital heart disease, heart valve disease, and other cardiovascular diseases. In both groups, a 256-layer spiral CT examination was performed. A pulmonary vein scanning protocol was applied to the patients with atrial fibrillation, and this can perform normal coronary angiography and exclude those with cardiovascular diseases such as congenital heart disease and valvular heart disease. The purpose of this study is to investigate the anatomical changes of the left atrium and its adjacent structures by applying the 256 nm spiral CT imaging to visualize the left atrium and its adjacent structures and by applying the MPR technology, VR technology, and simulation endoscope techniques.

## 1. Introduction

Antiarrhythmic drugs are the traditional treatment for arrhythmias, but they are less effective and have more side effects [1]. In particular, since the publication of CAST trial results in the late 1980s, the arrhythmogenic effect of antiarrhythmic drugs has been widely recognized, i.e., antiarrhythmic drugs may induce or aggravate arrhythmias while treating arrhythmias. 1986 saw the first application of radiofrequency energy ablation in basic experiments, and the reports of radiofrequency ablation in canine hearts were also published. It was possible to achieve ablation by changing the temperature and energy [2]. In 1986, the first application of radiofrequency energy ablation was performed in basic experiments, and the first report of radiofrequency ablation in the canine heart was published. After the publication of these two studies, the radiofrequency ablation of the catheters gradually gained attention and developed rapidly, and it was soon applied to humans, ushering in the era of the radiofrequency ablation of cardiac arrhythmias. Radiofrequency ablation is a form of electric current that can be converted into electrical energy. It mainly produces an impedance thermal effect on the local tissues, evaporating and drying the water in cardiomyocytes, forming a small, well-defined circular or oval coagulative necrosis to achieve the purpose of ablation [3]. After more than 20 years of development, improvement, and clinical popularity, radiofrequency ablation has gradually become the main way of the radical treatment of cardiac arrhythmias and the first-line clinical treatment modality [4]. It can cure a variety of arrhythmias, including atrial tachycardia, atrial tachycardia, paroxysmal ventricular tachycardia, early atrial fibrillation, and atrial tachycardia. In the treatment of some arrhythmias, radiofrequency ablation can be the method of choice. At the same time, the development of radiofrequency ablation has also enriched and expanded the understanding of arrhythmia, i.e., “learning by burning” [5].

The article "Spiral Computed Tomography in the Quantitative Measurement of the Adjacent Structure of the Left Atrial Appendage in Patients with Atrial Fibrillation" was retracted in 2023. Reasons: signs of a paper mill; suspected computer-generated content; unreliable results or conclusions; lack of ethics approval or compliance.

The clinical electrophysiology practice has found that some atrial arrhythmias, such as atrial tachycardia, or ventricular arrhythmias, such as ventricular premature and ventricular tachycardia, are more difficult to be successfully ablated using a conventional endocardium, while they can be successfully ablated in the vicinity of the aortic sinus [6]. However, the anatomy of the aortic root is very complex, and a full understanding of the adjoining and anatomical structures of the aortic root is very important for the successful ablation of arrhythmias and the reduction of complications. Basic studies have found that the aortic sinus includes three sinuses: the noncoronary sinus (NS). More commonly, the ablation of the noncoronary sinus can eradicate some right atrial tachycardia, and the ablation of the left coronary sinus orifice region can eradicate some left ventricular idiopathic/ventricular premature/ventricular tachycardia [7]. This led us to consider how the aortic sinus and its adjoining structures become arrhythmogenic substrates and how the ablation of the aortic sinus and its adjoining structures can eradicate arrhythmias. It relies on the further understanding of the anatomy of the aortic sinus and its frequent adjacent tissues. At present, there are a few studies in China and abroad, and most of them focus on animal observation, autopsy, or visual observation during cardiac surgery, which lacks clinical guidance [8]. This is achieved by the slip ring technology and a continuous flat movement of the scanning bed [9]. The subjects underwent selective pulmonary venography (CPV) during the subsequent ablation of atrial fibrillation to measure the entrance diameter of each pulmonary vein, and these data were used as a control group [10]. Patients with a positive contrast allergy test, patients with decompensated neurological insufficiency, patients with severe cardiac and renal insufficiency (creatinine >10 *μ*mol/L), and patients who were unable to cooperate with poor breath-holding during the respiratory training were excluded from the pulmonary venous and left atrial angiography using a 320-slice spiral CT; all patients signed an informed consent form before the examination. If a patient had a pulmonary vein variant detected after successful examination, that patient was also excluded [11]. All patients were required to fast for at least 6 h before performing the pulmonary venous left atrial angiography. Then, venous access was established and an indwelling cannula was placed in the anterior elbow vein.

The article "Spiral Computed Tomography in the Quantitative Measurement of the Adjacent Structure of the Left Atrial Appendage in Patients with Atrial Fibrillation" was retracted in 2023. Reasons: signs of a paper mill; suspected computer-generated content; unreliable results or conclusions; lack of ethics approval or compliance.

The patient's weight is routinely measured for an accurate contrast dosage, and an electrocardiogram is performed. The patient should be placed in a supine position with the scanning direction on the front of the foot. The electrodes should be placed correctly in the standard position with the ECG leads connected and the ECG signal confirmed to be received before the scan; the patient is then trained to breathe to minimize the artifacts caused by the respiratory movements so that he can cooperate with the examination.

## 2. Related Work

94% of ectopic electrical activity originates from the pulmonary veins. Abnormal extracardiac potentials are the main cause of paroxysmal atrial fibrillation [12]. Clinically, radiofrequency ablation for pulmonary vein isolation is currently an effective treatment for patients in whom antiarrhythmic drugs are ineffective. However, because of the complex anatomical structure of the pulmonary veins, individual variability, and more variability, the accurate placement of the marker device and the ablation effect can be affected by many of these factors [13]. However, different imaging techniques have their advantages and disadvantages. With the continuous updating of the CT imaging equipment, CT angiography has been widely used for noninvasive vascular imaging before the ablation of atrial fibrillation [14].

Ventricular arrhythmias are one of the more common critical illnesses in clinical work. There are many types of ventricular arrhythmias, including ventricular tachycardia, ventricular fibrillation, premature ventricular contractions, ventricular flutter, and supraventricular arrhythmias, such as atrial fibrillation, supraventricular tachycardia, and preexcitation syndrome [15]. Most arrhythmias are associated with heart diseases. However, some patients without organic heart disease also develop ventricular arrhythmias. Such cases account for approximately 10% of the patients with arrhythmias and idiopathic ventricular arrhythmias. Atrial fibrillation is the most common persistent arrhythmia in clinical practice, and its prevalence increases with age, seriously affecting people's health. In recent years, the incidence of AF has been increasing significantly with age. The number of patients with AF is gradually increasing as the number of aging people in China further increases. Its high morbidity and disability rate have caused more and more clinical; epidemiological statistics found that the adult prevalence of AF in China is approximately 0.77%. There are approximately more than 8 million patients with AF, and the incidence is similar to that of Western countries [16]. The current treatment strategy for idiopathic ventricular arrhythmias is guided by the severity of the patient's clinical symptoms and the risk of sudden death. Although the use of antiarrhythmic drugs can reduce the patient's symptoms to some extent, the effect is less satisfactory in reducing the patient's risk of sudden death. The placement of cardioverter-defibrillators in the patients can effectively terminate and reduce the mortality rate to an extent, but only for some. The cardioverter-defibrillator is effective in terminating and reducing mortality, but only in certain populations, and it is not effective in reducing arrhythmias [17].

The article "Spiral Computed Tomography in the Quantitative Measurement of the Adjacent Structure of the Left Atrial Appendage in Patients with Atrial Fibrillation" was retracted in 2023. Reasons: signs of a paper mill; suspected computer-generated content; unreliable results or conclusions; lack of ethics approval or compliance.

Multiple abnormal potential trigger points in the pulmonary veins play an important role in the development and progression of AF. The myocardial tissue of the left atrium extends into the outer layer of the pulmonary vein wall, which, in turn, forms a myocardial sleeve. This extended myocardial sleeve is the release point for the abnormal potential activity, and it has been demonstrated that approximately 94% of the abnormal potential triggers are from the pulmonary veins [18]. Supraventricular arrhythmias, such as atrial fibrillation, generally have a long history, significant myocardial fibrosis, more complications, high risk of stroke with drug therapy, poor efficacy, and arrhythmogenic effects with the long-term application of antiarrhythmic drugs in such patients. Therefore, there is much interest in the clinical effectiveness and safety of transcatheter ablation for the treatment of AF [19]. Current studies suggest that most cases of paroxysmal AF are triggered or driven by the extracardiac abnormal potential sites and the pulmonary veins are the most common sites of origin for such arrhythmias that often cause paroxysmal AF. Therefore, it is believed that the effective treatment of paroxysmal AF can be achieved by implementing the electrical isolation of the pulmonary veins to terminate the ectopic potential generation.

The radiofrequency ablation of the pulmonary veins causing arrhythmia can lead to the eradication of paroxysmal atrial fibrillation [20]. The purpose of the catheter radiofrequency ablation of atrial fibrillation is to form an effective electrical isolation between the pulmonary veins and the atria. The necessary tool for the electrical isolation of the pulmonary veins in radiofrequency ablation, the annulus, is the marker electrode, which is placed at the entrance of the pulmonary veins via a catheter after performing an atrial septal puncture. The annular plane is placed parallel to the entrance of the pulmonary veins. The most used electrode diameters in clinical practice are 1.5 cm and 2.0 cm, and the diameter of the calibrated electrode chosen during the procedure should be slightly larger than the diameter of the pulmonary vein to be ablated [21]. The normal anatomy of the pulmonary veins has four pulmonary veins, and when anatomical variations occur, the number of pulmonary veins varies. A normal pulmonary vein's anatomy accounts for about 70% of the total in the studied population while the pulmonary vein's anatomical variations occur in about 19–30% of the normal population. Different pulmonary vein branches in the same patient and the same pulmonary vein branch in different patients have very different morphology, diameter, angle, and branches at the entrance of their pulmonary veins. There are also differences in the angle and branch of the same pulmonary vein in different patients.

## 3. Helical Tomography of Structures Adjacent to the Left Heart Ear

### 3.1. Left Atrial Angiography

A total of 105 subjects were selected who underwent the 320-slice spiral CT pulmonary vein and left atrial angiography in the radiology department from November 2017 to March 2021. 58 were male and 47 were female. The mean age was 58 ± 12 years. The patients with positive contrast allergy test, patients with decompensated neurological insufficiency, patients with severe cardiac and renal insufficiency (creatinine >10 *μ*mol/L), and patients with poor breath-holding ability to cooperate were excluded. All patients signed an informed consent form before the examination. The patients were also excluded if the pulmonary vein variation was detected after a successful examination.

The article "Spiral Computed Tomography in the Quantitative Measurement of the Adjacent Structure of the Left Atrial Appendage in Patients with Atrial Fibrillation" was retracted in 2023. Reasons: signs of a paper mill; suspected computer-generated content; unreliable results or conclusions; lack of ethics approval or compliance.

All patients were required to fast for at least 6 h before performing the pulmonary venous left atrial angiography. Then, intravenous access was established with an indwelling cannula placed in the anterior elbow vein. If the patient's heart rate is > 70 beats/min, the patient should be advised to breathe steadily and be reassured with words to keep the patient as calm as possible. The heart rate should be controlled to less than 70 beats per minute.

The patient should be placed in a supine position with the scanning direction in the direction of the head of the foot. Before scanning, the electrodes should be placed correctly with the ECG leads connected in the standard position and the ECG signal should be confirmed. Toshiba AQULION ONE TSX-304A 320-slice spiral CT with cardiac gating technology was used. The scan was performed in a calm breathing state with breath-holding from 5 mm below the tracheal bifurcation to 10 mm below the diaphragmatic surface of the heart using a whole-heart volume scan. The subject was placed in the supine position with the foot and head orientation to confirm that the ECG signal was received as shown in Figure 1; a Toshiba AQULION ONE TSX-304A 320-row spiral CT was used to perform the scan using cardiac gating technology. The pulmonary vein and left atrial CTV scan sequences were selected and the sure start software intelligently triggered the scan with the trigger point range set at the level of the root of the ascending aorta and a trigger threshold of 320 HU. The scan was performed in a calm breathing state with breath-holding from 5 mm below the tracheal bifurcation to 10 mm below the diaphragmatic surface of the heart using the whole-heart volume scanning. The tube voltage was 100 kV, tube current was 600 mA, full heart volume acquisition range was 320 rows × 0.5 mm, frame speed was 350 ms, and the rotational scan time was 140 ms. The area of interest was set in the left atrium at the mitral level and the enhancement scan was automatically triggered. The average scan time was 2.5 s. The resulting data were reconstructed at 75% of the RR interval. The images are uploaded to a postprocessing workstation and reconstructed using postprocessing techniques, such as multiplanar reconstruction, volume reproduction, maximum density projection, and simulated endoscopy, which showed a long-axis image of the left atrium and pulmonary veins, with the pulmonary vein trunk intact. The patients undergoing atrial fibrillation ablation should have a clinical diagnosis of atrial fibrillation that has failed to respond to the antiarrhythmic drug therapy.

The article "Spiral Computed Tomography in the Quantitative Measurement of the Adjacent Structure of the Left Atrial Appendage in Patients with Atrial Fibrillation" was retracted in 2023. Reasons: signs of a paper mill; suspected computer-generated content; unreliable results or conclusions; lack of ethics approval or compliance.

### 3.2. Spiral Tomography-Based Ablation of Atrial Fibrillation

The subjects were patients with clinically diagnosed atrial fibrillation for whom antiarrhythmic drug therapy had failed. The patients with severe cardiac insufficiency and untreated valvular disease, pulmonary hypertension, coagulation abnormalities, severe hyperthyroidism, and multiorgan failure of the liver and kidneys were excluded, preoperatively. All patients signed an informed consent form and a surgical protocol. The patients should be admitted for routine investigations: screening for infectious diseases, laboratory tests (blood and urine routine, coagulation function, thyroid function, liver and kidney function, electrolytes, NT-pro BNP), and cardiac echocardiography to understand the left ventricular systolic function, clarify the size of each atrium and left atrial diameter, routine electrocardiogram, monitoring of 24-hour heart rate by 24-hour ambulatory electrocardiogram, and pulmonary CT or X-ray chest orthopantomogram. Pulmonary CT or X-ray chest frontal and lateral radiographs were performed for routine pulmonary examination. The patients taking warfarin INR at the preoperative level should be tested for intraoperative heparin dosage that must be reduced appropriately. The patients taking new anticoagulant drugs should discontinue the drugs 12–24 hours before the surgery. Intraoperative heparin dosage (80–100 *μ*/kg) should be accurate and adjusted in a timely manner based on intraoperative clotting time.

The patient is placed flat on the angiographic C-arm bed and the position of the patient's heart is confirmed to be in the center of the C-arm bulb before the procedure. The left femoral vein and the left subclavian vein are punctured, and the target catheter is placed into the coronary sinus and the right ventricle, respectively. The atrial septal puncture needle is fed through the left femoral vein catheter. The septum is penetrated and contrast is sprayed to visualize the image of the left atrium. Heparin (100 *μ*/kg) is injected when the septal puncture is completed, and additional heparin (1000 *μ*/hour) is added intraoperatively to prevent thrombosis. The catheter is fed through the femoral vein, pointed at the target vein, and after sufficient venting, a high-pressure syringe is connected and the contrast agent (1.2 ml/kg) is injected. The C-arm rotational imaging mode is selected with the tube ball in the starting position and the delayed acquisition time at 0. After the high-pressure syringe triggers the linkage to inject the contrast agent, the images are acquired by rotating the patient at a rate of 30 frames/second with a rotation time of 4-5 seconds. The catheter is perfused with cold saline via the Swartz sheath, and the loop electrode is delivered to the left atrium.

The article "Spiral Computed Tomography in the Quantitative Measurement of the Adjacent Structure of the Left Atrial Appendage in Patients with Atrial Fibrillation" was retracted in 2023. Reasons: signs of a paper mill; suspected computer-generated content; unreliable results or conclusions; lack of ethics approval or compliance.

### 3.3. Quantitative Results of the Main Left Auricular Adjacent Connection Structure

The observation and analysis of MSCT imaging data of 100 patients revealed that there was a connection structure between the three sinus walls of the aortic sinus (coronary sinus, left coronary sinus, and right coronary sinus) and atrium/ventricle (coronary sinus), as shown in Figure 2. The number of cases connected and the percentage of the total number of connected cases were as follows: 48 patients (21.82%) had aortic sinus-right ventricle tissue connections, 23 patients (10.45%) had aortic sinus -left ventricle tissue connections, 20 patients (9.09%) had aortic sinus-right atrium tissue connections, 25 patients (11.36%) had the right coronary sinus-right ventricular tissue connection, 23 patients (10.45%) had the right coronary sinus-left ventricular tissue connection, 16 patients (7.27%) had the left coronary sinus-right ventricular tissue connection, 20 patients (9.09%) had the left coronary sinus-left ventricular tissue connection, and 45 patients (20.45%) had the left coronary sinus-left ventricular tissue connection. No connection structure was found between the coronary sinus and the ventricle. The most common connection was between the coronary sinus and the atrium. After x2 analysis, there was a significant difference in the connection between the left coronary sinus, the right coronary sinus, and the coronary sinus and peripheral tissues (*P* < 0.01). Thus, according to the connection structure, they were divided into groups without coronary sinus, left coronary sinus group, and right coronary sinus group. The connections were defined as the presence of a contact between the aortic sinus and the endocardia of the atrial ventricular tissue or of tissue connections. Figure 2 shows the presence of a connection to the peripheral atrium and ventricle from the aortic sinus under 3D reconstruction. The lower table shows the number of cases where the aortic sinus is connected to the surrounding tissue and the lower X2 is applied. Analyze whether there is a difference.

The aortic root was reconstructed by the MSCT software, scanned from 10 levels. The distance between the left coronary sinus without a right ventricular sinus and right coronary sinus and atrial/ventricular connection structure was measured and averaged. As shown in Figure 3, the distance between the coronary sinus and the atrium: the distance between the coronary sinus and the right atrium was significantly smaller than the distance between the coronary sinus-left atrium (1.77 ± 0.85 mm versus 2.22 ± 0.92 mm, *P* < 0.01). For the distance between the left coronary sinus and the atrium/ventricle, the left coronary sinus-right ventricle distance is significantly greater than the left coronary sinus-left coronary sinus and the left coronary sinus-left ventricle distance. We compared the left coronary sinus-left ventricle distance and the left coronary sinus-left ventricle distance (*P* < 0.01). For the right coronary sinus atrial/ventricular distance, the right coronary sinus-right ventricle distance is significantly smaller than the right coronary sinus-right ventricle distance. The distance between the coronary sinus and the right coronary sinus-left ventricle was significantly greater than that of the right coronary sinus and left ventricle (*P* < 0.05). However, there was no significant difference between the right coronary sinus and the right ventricle and the right coronary sinus and the left ventricle.

The article "Spiral Computed Tomography in the Quantitative Measurement of the Adjacent Structure of the Left Atrial Appendage in Patients with Atrial Fibrillation" was retracted in 2023. Reasons: signs of a paper mill; suspected computer-generated content; unreliable results or conclusions; lack of ethics approval or compliance.

There were tissue connections between the aortic sinus and the atria and ventricles, which could be fatty connections, fibrous connections, etc.: the aortic sinus-right atrium connection was present in 48 patients, the aortic sinus-left atrium connection in 23 patients, the right coronary sinus-right atrium connection in 20 patients, the right coronary sinus-right ventricle connection in 25 patients, the right coronary sinus-left ventricle connection in 23 patients, the left coronary sinus-right ventricle connection in 16 patients, the left coronary sinus-left ventricle connection in 20 patients, and the aortic sinus-right ventricle connection in 45 patients. The right ventricular connection was present in 23 patients, the left coronary sinus-right ventricular connection was present in 16 patients, the left coronary sinus-left atrial connection was present in 20 patients, and the left coronary sinus-left ventricular connection was present in 45 patients. The right coronary sinus-right ventricle was significantly shorter than the right coronary sinus-right atrium and right coronary sinus-left ventricle distances (1.85 ± 0.93 mm vs. 2.16 ± 0.99 mm, 2.01 ± 0.77 mm, *P* < 0.05), respectively, and the right coronary sinus-right atrium distance was significantly greater than the right coronary sinus-left ventricle (*P* < 0.05).

## 4. Experiments and Results Analysis

### 4.1. Anatomical Features of the Left Auricular Connection

The left coronary sinus is located posteriorly above the right ventricular outflow tract, adjacent to the root of the pulmonary artery and the left atrium. The right coronary sinus is located above the atrioventricular junction, posterior to the area of the bundle of Hitchcock and is connected to the atrioventricular node, adjacent to the right ventricle and right atrium. In this study, the right and left coronary sinuses were found to be connected mainly to the ventricular tissue, and the left coronary sinus was most commonly connected to the left ventricle, with 45 (20.45%) connected cases. Can it be stated that the ventricular arrhythmias associated with the aortic sinus can be successfully ablated by the ablation of the left coronary sinus? 44 patients with idiopathic ventricular arrhythmias associated with the aortic sinus (including ventricular premature and ventricular tachycardia) were studied, and the results showed that of all 44 patients, 24 patients were successfully ablated in the left coronary sinus, 14 patients were successfully ablated in the right coronary sinus, only 1 patient was successfully ablated in the noncoronary sinus, and 5 patients had a successful ablation in the left and right coronary sinus junctions. It showed that ventricular arrhythmias associated with the aortic sinus were mostly seen in the left coronary sinus. However, the relationship between the aortic sinus and the interventricular junction is poorly studied. Most cases are reported on a case-by-case basis, and there is a lack of relevant imaging evidence.

The article "Spiral Computed Tomography in the Quantitative Measurement of the Adjacent Structure of the Left Atrial Appendage in Patients with Atrial Fibrillation" was retracted in 2023. Reasons: signs of a paper mill; suspected computer-generated content; unreliable results or conclusions; lack of ethics approval or compliance.

In the ablation of frequent ventricular premature or ventricular tachycardia associated with the aortic sinus, ventricular arrhythmias originating in the left coronary sinus were the most common. The analysis of 7 cases of frequent ventricular premature or ventricular tachycardia associated with the aortic sinus led to the conclusion that 5 of them were successfully ablated in the left coronary sinus and the remaining 2 in the right coronary sinus. The mean distance from the left coronary sinus to the left trunk opening was 12.2 ± 3.2 mm. 12 cases of ventricular tachycardia were successfully ablated in the aortic sinus, and 9 cases were successfully ablated in the left coronary sinus. The majority of ventricular tachycardias were successfully ablated in the left coronary sinus, which may be related to the closer proximity of the left coronary sinus to the left ventricle in this study. Histological studies also revealed crescentic myocardial tissue connections between the aortic sinuses, especially the left and right coronary sinuses, and the right and left ventricular myocardium. These connecting structures may be the extensions of the ventricular myocardium to the aortic sinus and may be the ectopic points of origin for ventricular arrhythmias originating from the aortic sinus. In this study, the presence of connecting structures in the right coronary sinus-right ventricle, right coronary sinus-left ventricle, left coronary sinus-right ventricle, and left coronary sinus-left ventricle was confirmed from an imaging perspective by applying MSCT. These connecting structures may serve as conduction channels between the aortic sinus-ventricle, making the aortic sinus a substrate for ventricular arrhythmias. Consistent with the results of previous studies, the present study showed that the left coronary sinus-left ventricle connection was the most common, which could explain the predominance of the aortic sinus-related ventricular arrhythmias associated with the left coronary sinus as shown in Figure 4. In addition, during the ablation of the left and right coronary sinus, to prevent complications in addition to the strict control of RF energy, it is also important to clarify the anatomical relationship between the coronary artery opening and the ablation target. Many scholars believe that the ablation of the aortic sinus should ensure a distance greater than 1 cm from the left and right coronary orifices, but others believe that this distance of 5–8 mm is considered safe. Therefore, most centers at home and abroad should routinely perform coronary angiography to place contrast catheters before the ablation of the left and right coronary sinuses to mark the coronary openings and avoid coronary opening or intracoronary discharge ablation to reduce the occurrence of complications such as coronary syndrome. The coronary sinus-right atrial distance was significantly smaller than the coronary sinus-left atrial distance (1.77 ± 0.85 mm vs. 2.22 ± 0.92 mm, *P* < 0.05). The left coronary sinus-right ventricular distance was significantly greater than the left coronary sinus-left atrial distance and the left coronary sinus-left ventricular distance (2.66 ± 0.57 mm vs. 2.05 ± 0.91 mm, 1.90 ± 0.45 mm, *P* < 0.05).

The article "Spiral Computed Tomography in the Quantitative Measurement of the Adjacent Structure of the Left Atrial Appendage in Patients with Atrial Fibrillation" was retracted in 2023. Reasons: signs of a paper mill; suspected computer-generated content; unreliable results or conclusions; lack of ethics approval or compliance.

### 4.2. Comparison of Information between Atrial Fibrillation Group and Control Group

In this study, a total of 174 patients, including 94 patients with atrial fibrillation and 80 patients with normal rhythm, included a comparison of age, gender, height, and weight among the groups of atrial fibrillation and nonatrial fibrillation (*P* < 0.05), while the body weight was higher in the atrial fibrillation group than in the nonatrial fibrillation group (*P* < 0.05). The difference in gender and height was statistically significant (*P* > 0.05). The incidence of male patients with atrial fibrillation was significantly higher than that of the female patients. The ratio of left atrial fibrillation was different between atrial fibrillation and control. In the atrial fibrillation group, we considered the number of cases of type A I, type A II, type B, and type C and the proportions of the cases were 10 (10.6%), 38 (40.4%), 38 (40.4%), and 8 (8.5%), respectively. There were 12 (15.0%), 51 (78.8%), 8 (10.0%), and 9 (11.3%) in the number of cases of type A I, type A II, type B, type C in nonatrial fibrillation group, respectively. As shown in Figure 5, the percentages of type A I, type A II, and type C were lower in the atrial fibrillation group than in the control group, and the percentage of type B was higher than the control group.

Quantitative analysis of the left upper pulmonary vein and the mitral ring atrial fibrillation group and nonatrial fibrillation group was performed by comparing the minimum distance from the left atrium to the left upper pulmonary vein and left atrial branch, the width of the crista, the upper margin of the left atrium, the middle edge, the lower edge, and the opening of the left atrium. The data were compared between the two groups (Figure 6). The minimum distance from the left atrium to the upper pulmonary vein and the distance from the opening of the left atrium to the opening of the left upper pulmonary vein and the mitral ring increased in the atrial fibrillation group in comparison with nonatrial fibrillation. In the atrial fibrillation group, the minimum distance from the left atrium to the left gyral branch, the top length of the left atrium, and the width of the top of the apex were reduced in comparison with the nonatrial fibrillation group (*P* < 0.05).

The left auricle is generally located in the atrioventricular sulcus of the free wall of the left atrium and has a complex relationship with the surrounding adjacent structures. The anterior wall is close to the proximal coronary artery gyrus and travels upward close to the root of the pulmonary artery. The left auricle and the left auricular crest are highly variable, and some studies have shown that an excessive ablation in the left auricular crest has the risk of causing pulmonary vein stenosis. There are also case reports of patients with atrial fibrillation in whom the ablation of the base of the left auricle was performed, improperly resulting in a perforation, and possibly, it resulted in a left gyral branch-left atrial fistula. A multilayer spiral CT examination has an obvious superiority in observing the display of cardiac structures. Coronary CT angiography (CTA) is mostly used in clinical practices to observe the cardiovascular lesions, while pulmonary vein scanning parameters are mostly used in patients with atrial fibrillation.

A 256-layer spiral CT can clearly observe the anatomical structure of the heart by a powerful image posttreatment technique. It follows the understanding of certain anatomical structures of the left atrium and pulmonary veins before the surgery, atrial fibrillation, and follow-up of the presence of pulmonary vein stenosis after RF ablation. The incidence of atrial fibrillation was high in the middle-aged and elderly subjects. The average age of the subjects in both experimental and control groups was higher in this study, 57.46 ± 11.68 and 56.10 ± 7.83 years in the atrial fibrillation group. As shown in Figure 7, there was no significant difference in the age between the two groups in the nonatrial fibrillation group (*P* < 0.05). The weight of patients in the atrial fibrillation group was found to be an independent risk factor for the development of atrial fibrillation by the nonatrial fibrillation group and follow-up study. The high-frequency ablation therapy may exacerbate the symptoms and the load of atrial fibrillation. The frequency of radiofrequency ablation therapy is also suitable for obese patients.

The article "Spiral Computed Tomography in the Quantitative Measurement of the Adjacent Structure of the Left Atrial Appendage in Patients with Atrial Fibrillation" was retracted in 2023. Reasons: signs of a paper mill; suspected computer-generated content; unreliable results or conclusions; lack of ethics approval or compliance.

In addition, the results of the study found that the crest length and the width of the superior margin of the crest were shorter and statistically different in the patients with atrial fibrillation than in the control group. The patients with atrial fibrillation should pay attention to the morphology and diameter of the left auricular crest when performing the circumferential pulmonary vein spot isolation to avoid damage to other structures or tissues during the operation and to make the scope of the procedure more precise. The left anterior descending coronary and gyral branches are very close to the left auricle or its opening and are susceptible to trauma during percutaneous device implantation, especially when the device is greater than 20% to 40% OS. The results of this study show that the minimum distance from the left auricle to the left gyral branch is small in patients with atrial fibrillation compared to controls, and the majority of the patients have a close distance between the base of the left auricle and the gyral branch of the coronary artery. When performing the radiofrequency ablation of the left auricle, the operator needs to be more careful to prevent the perforation of the left auricle with damage to the left gyral branch because of improper operation. The operator has to be careful to not cause a left auricle-left gyral branch fistula. There is also a risk of compression of the left gyral branch by an oversized blocking device when performing a left auricular occlusion as shown in Figure 8. This study mainly focused on patients with and without atrial fibrillation. Other cardiovascular system diseases were not included in the grouping criteria of the atrial fibrillation group. It may produce errors in the experimental results, but this can be a direction for future studies to understand the pathogenesis of atrial fibrillation more carefully.

The article "Spiral Computed Tomography in the Quantitative Measurement of the Adjacent Structure of the Left Atrial Appendage in Patients with Atrial Fibrillation" was retracted in 2023. Reasons: signs of a paper mill; suspected computer-generated content; unreliable results or conclusions; lack of ethics approval or compliance.

Atrial fibrillation, which is common in the elderly, can be classified according to the characteristics of episodes as paroxysmal (lasting <7 hours, self-resetting rate), persistent (meaning lasting >7d, generally not self-resetting), and permanent (failure of resetting to maintain sinus rhythm or no indication for resetting) atrial fibrillation. Irregular atrial fibrillation and ventricular rate derangement can cause a series of clinical symptoms such as dyspnea, palpitations, chest tightness, etc. In severe cases, it can cause heart failure and stroke. A large number of studies have shown that the left auricle (LAA) is closely related to the occurrence and development of atrial fibrillation. In 90% of the patients with atrial fibrillation, the cardiogenic thrombus forms in the left auricle, the atria lose their rhythmic contraction, the pumping capacity decreases, and the ability of the left auricle to drain the blood decreases, making it easy to form a thrombus. In addition, recent studies have found that the left heart ear can act as a trigger point for atrial arrhythmias. To treat atrial fibrillation, restore the normal rhythm of the atria, prevent the formation of thrombus and help patients improve their quality of life, pharmacological and surgical treatments are mostly used in clinical practices.

At present, radiofrequency ablation and left ear occlusion are a new trend of development that is mostly applied to treat patients with atrial fibrillation for whom drug therapy is ineffective. Radiofrequency ablation can ablate the rapid conduction or specific areas of cardiomyocytes in the patients with atrial fibrillation to reduce the symptoms of atrial fibrillation. The left ear occlusion is used to occlude the left ear by selecting a suitable occluder, which is mostly used to prevent the formation of left ear thrombus in the patients with atrial fibrillation or to prevent the dislodgement of the formed thrombus to reduce the risk of ischemic stroke. The implementation of both procedures requires precise observation and measurement of the left ear and its surroundings. Therefore, the quantitative study of the anatomy and function of the left auricle in the patients with atrial fibrillation can provide an objective imaging basis for the clinical treatment of patients with atrial fibrillation by initially exploring the clinical significance of the left auricle on the development and progression of atrial fibrillation. With the advancement of technology, multilayer spiral CT (MSCT) is widely used in various clinical examinations and has its unique advantages in diagnosing cardiovascular diseases and evaluating the anatomical structure of the heart. The images obtained from MSCT are of high quality and can evaluate the anatomical structure and function of the heart more objectively using various postprocessing techniques.

The article "Spiral Computed Tomography in the Quantitative Measurement of the Adjacent Structure of the Left Atrial Appendage in Patients with Atrial Fibrillation" was retracted in 2023. Reasons: signs of a paper mill; suspected computer-generated content; unreliable results or conclusions; lack of ethics approval or compliance.

## 5. Conclusion

The purpose of this study is to investigate the anatomical changes of the left atrium and its adjacent structures by applying the 256 nm spiral CT imaging to visualize the left atrium and its adjacent structures and by applying the MPR technology, VR technology, and simulation endoscope techniques. This has a large clinical value in the preoperative evaluation of patients with atrial fibrillation. It can provide an objective morphological reference of radiofrequency ablation and left atrial obstruction in patients with atrial fibrillation. In the quantitative CT study of 612 patients, with or without AF, the left auricular opening was found to be oval (68.9%), pedunculated (10%), triangle (7.7%), and tear drop (7.7%). It is suggested that the diameter calculated from the circumference of the left auricular opening of the MSCT image is more reliable than directly measuring the diameter and area of the left ear opening. In most cases, it is difficult to accurately measure the diameter of the left ear opening because the plane of the left auricular opening obtained by tee or MRCT may not be parallel to the true left ear opening even if MDCT multiplane reconstruction is used. As the shape of the opening is very irregular, it is difficult to reconstruct the cross-section of the left ear opening. The patient was lying flat on the angiography bed, and the preoperative position of the patient's heart was confirmed to be in the central region of the C-arm tube bulb. The left femoral vein and the left subclavian vein were punctured, and the catheter was placed into the coronary sinus and the right ventricle, respectively.

## Figures and Tables

**Figure 1:** Spiral tomographic process under atrial fibrillation.

**Figure 2:** Analysis of aortic sinus connection to atrial or ventricular tissue.

**Figure 3:** Analysis of variance for the left atrial distance row.

**Figure 4:** *χ* ^2^ analysis of the number of cases in which the aortic sinus was connected to the atrium and ventricle.

**Figure 5:** Comparison of clinical data between the atrial fibrillation group and control group.

**Figure 6:** Comparison of left atrial crest fractions in the atrial fibrillation group and control group.

**Figure 7:** Atrial fibrillation load in the atrial fibrillation group versus the control group.

**Figure 8:** Variation in left auricular-left gyral distance.

The article "Spiral Computed Tomography in the Quantitative Measurement of the Adjacent Structure of the Left Atrial Appendage in Patients with Atrial Fibrillation" was retracted in 2023. Reasons: signs of a paper mill; suspected computer-generated content; unreliable results or conclusions; lack of ethics approval or compliance.

## Data Availability

The data used to support the findings of this study are available from the corresponding author upon request.
